# Super Resolution Image Visual Quality Assessment Based on Feature Optimization

**DOI:** 10.1155/2022/1263348

**Published:** 2022-06-20

**Authors:** Shu Lei, Huang Zijian, Yan Jiebin, Fei Fengchang

**Affiliations:** ^1^School of Information Technology, Jiangxi University of Finance and Economics, Nanchang 330032, China; ^2^College of Modern Economics and Management, Jiangxi University of Finance and Economic, Nanchang 330032, China

## Abstract

Most existing no-referenced image quality assessment (NR-IQA) algorithms need to extract features first and then predict image quality. However, only a small number of features work in the model, and the rest will degrade the model performance. Consequently, an NR-IQA framework based on feature optimization is proposed to solve this problem and apply to the SR-IQA field. In this study, we designed a feature engineering method to solve this problem. Specifically, the features associate with the SR images were first collected and aggregated. Furthermore, several advanced feature selection algorithms were used to sort the feature sets according to their importance, and the importance matrix of features is obtained. Then, we examined the linear relationship between the number of features and Pearson linear correlation coefficient (PLCC) to determine the optimal number of features and the optimal feature selection algorithm, so as to obtain the optimal model. The results showed that the image quality scores predicted by the optimal model are in good agreement with the human subjective scores. Adopting the proposed feature optimization framework, we can effectively reduce the number of features in the model and obtain better performance. The experimental results indicated that SR image quality can be accurately predicted using only a small part of image features. In summary, we proposed a feature optimization framework to solve the current problem of irrelevant features in SR-IQA, and an SR image quality assessment model was proposed consequently.

## 1. Introduction

Image super-resolution (ISR) refers to the recovery of a high-resolution image from a low-resolution image. Early ISR methods are mainly based on interpolation [1–3], where ISR is regarded as a signal resampling problem [4]. Similar to other tasks such as semantic segmentation [5], depth estimation [6], and point cloud analysis [7], ISR plays an important role in the development of image processing and computer vision. In recent years, with the popularity of machine learning, most SR algorithms proposed in literature are based on machine learning. Their merit is that they can learn additional information from existing samples. Dong et al. [8] used a convolutional neural network (CNN) to simulate the encoding and decoding of dictionary-based ISR. Ding *et al.* [9] imitated the behavior of sparse coding by inserting a subnetwork and embedded sparse constraints into CNN. Johnson et al. [10] used trained VGGNet [11] to extract SR features related to visual perception. Generally, PSNR and SSIM [12] are applied as the standards of SR image quality assessment (IQA). However, the work of [13] shows that PSNR and SSIM cannot accurately predict the quality of SR images.

In order to solve the above problems, Zhou et al. [4] proposed a full-reference (FR) super resolution (SR)-IQA method, which is more suitable for SR-IQA than other FR methods. Nevertheless, source images are often missing in practical applications. So, the FR IQA methods cannot meet the practical requirement well. No-referenced (NR) IQA based on Natural Scene Statistics (NSS) has achieved great success in IQA fields [14–16]. In [14], an NR-IQA method called BLINDS2 based on discrete cosine transform (DCT) is proposed. Mittal et al. [15] used local normalized brightness coefficients that are based on NSS to quantify image distortion and evaluate images quality. By studying real distorted images in different color spaces and transform domains, an NSS-based method was proposed to extract a series of features [16]. In recent years, several NR-IQA methods have been proposed. In [17], three types of statistical features are used to quantify artifacts and evaluate the quality of SR images. Considering that handcraft features cannot accurately quantify the degradation of SR images, Zhang et al. [18] used VGGNet to extract features of SR images first, then used a superposition regression framework to predict the SR image quality. The NR-SRIQA (no reference-super-resolution image quality assessment) method is realized by establishing the relationship between image depth feature and quality score. A no-reference perceptual quality assessment method is developed for JPEG coded stereoscopic images based on segmented local features of distortions and disparity [19], as well as the blockiness and the edge distortion within the block of images are evaluated in this method. Combining the color difference formula of CIEDE2000 and the printing industry standard for visual verification, Yang et al. [17] presented an objective color image quality assessment method correlated with subjective vision perception. In view of the defects of rough image segmentation and high spatial distortion rate in current sports video image evaluation methods, Fan et al. [20] proposed a sports video image evaluation method based on BP neural network perception. Aiming at the compression damage and transmission damage of leisure sports video, a video quality evaluation algorithm based on BP neural network (BPNN) was proposed in [21].

Despite all this, most of the above NR-IQA methods not only fail to consider the characteristic of SR images but also fail to find the balance between efficiency and performance. For example, the method proposed in [14] has a high computational complexity and costs a lot of time in feature extraction, which is unfriendly in real applications. Method proposed in [16] has excellent performance in SR tasks; however, the large number of features in this method brings high complexity. In addition, there are some methods that do not perform well on SR-IQA tasks, despite the low complexity. Moreover, most of the above NR-IQA methods may use redundant features, which degrades the performance of these methods. Therefore, it is very important to take a deep look at the features associated with SR-IQA tasks.

Inspired by the study of [22], a feature optimization framework is put forward in this paper, and an SR image quality assessment model is proposed consequently. First, the features related to the SR images are collected and aggregated to establish the initial feature set and model_a_. Second, this paper uses the popular feature selection algorithm to sort the initial feature set according to the importance of features. Each algorithm is performed 100 times and uses an assigned weight method to obtain the order of importance of the initial feature set. Then the linear correlation between the number of features and Pearson linear correlation coefficient (PLCC) is studied according to the importance matrix of features to determine the optimal number of features and the optimal feature selection algorithm. Besides, support vector machine (SVR) [23] is applied to learn a given number of features to build a model and predict the quality of SR images, and the PLCC between the predicted score and human subjective score is calculated. Finally, the optimal feature selection is determined by the linear correlation between PLCC and the number of features.

## 2. Related Works

### 2.1. NSS-Based IQA Models

The IQA model based on NSS is always the leading position in the field of IQA. These models assume that high-quality real-world photographic images that have been properly standardized and follow the statistical rules that change when distortion is introduced into the image. For example, Saad et al. [14] used the features of DCT coefficient changing with the introduction of distortion to predict image quality. Mittal et al. [15] used the features of mean subtracted contrast normalized (MSCN) coefficient changing with the introduction of distortion to establish IQA model, etc. All these changes can be captured by generalized Gaussian model.

Generalized Gaussian model [9, 10] has been widely used in the field of IQA. GGD is defined as

(1) $$\begin{array}{c} f\left(x;\alpha ,\sigma^{2}\right)=\frac{\alpha }{2\beta \Gamma \left(1/\alpha \right)}\exp\left(-{\left(\frac{\left|x\right|}{\beta }\right)}^{\alpha }\right),\\ \beta =\sigma \sqrt{\frac{\Gamma \left(1/\alpha \right)}{\Gamma \left(3/\alpha \right)}}, \end{array}$$

where Γ is gamma function, as defined below

(2) $$\begin{array}{c} \Gamma \left(a\right)=\int_{0}^{\infty }t^{a-1}e^{-t}dt\;a>0, \end{array}$$

where *α* controls the shape of the distribution and *σ* controls the variance. Asymmetric generalized Gaussian distribution (AGGD) is defined as

(3) $$\begin{array}{c} f\left(x,v,\sigma_{l}^{2},\sigma_{r}^{2}\right)=\left\{\begin{array}{cc} \frac{v}{\left(\beta_{l}+\beta_{r}\right)\Gamma \left(1/v\right)}\text{exp}\left(-{\left(\frac{-x}{\beta_{l}}\right)}^{v}\right) & x>0\\ \frac{v}{\left(\beta_{l}+\beta_{r}\right)\Gamma \left(1/v\right)}\text{exp}\left(-{\left(\frac{x}{\beta_{r}}\right)}^{v}\right) & x\geq 0 \end{array}\right., \end{array}$$

where

(4) $$\begin{array}{c} \beta_{l}=\sigma_{l}\sqrt{\frac{\Gamma \left(1/v\right)}{\Gamma \left(3/v\right)}},\\ \beta_{r}=\sigma_{r}\sqrt{\frac{\Gamma \left(1/v\right)}{\Gamma \left(3/v\right)}}. \end{array}$$

Among them, AGGD has three parameters, *v*, *σ*_*l*_, *σ*_*r*_, where *v* controls the shape of the distribution and *σ*_*l*_ and *σ*_*r*_ control the diffusion degree of left and right sides, respectively.

### 2.2. NR-IQA Model

Saad et al. [24] proposed a method which called “BLINDS-I” to predict image quality based on observing statistics of local DCT coefficients. In this model, the structural features and contrast features based on DCT were extracted at two scales, and then the image quality is predicted by probability prediction model; Mittal et al. [15] proposed an IQA model based on NSS spatial domain which called “BRISQUE,” they found that the brightness value of natural image presents a generalized Gaussian distribution. Based on this, the parameters of GGD and AGGD are used as features of distorted images, and then a SVR is applied to learn the features to predict image quality. The model does not calculate distortion specific features, such as ringing, blurring or blocking, but using local normalized brightness coefficient changes to calculate image quality. Based on BLINDS-I, Saad et al. proposed BLINDS-II by improving GGD and AGGD models [14]. In this model, GGD and AGGD model parameters are used as the features of distorted images. The model that is called “FRIQUEE” proposed by Deepti et al. [16] adopts a series of feature mapping methods, and they use the features that are sensitive to image quality, such as brightness feature (Luma) and Chroma feature (Chroma). Instead of quantifying the assumed image distortion, the model focuses on capturing the consistency or deviation of real-world image statistics to predict image quality; Ma et al. [17] designed three types of low-level statistical features in the spatial and frequency domains to quantify SR image artifacts. The model sets DCT, wavelet coefficient features in frequency domain, and sets PCA features in spatial domain, and then a two-stage regression model is used to predict the quality of SR images.

Some NR-IQA models are also represented by probability values or histograms. Li et al. [25] proposed a NR-IQA method called GWH-GLBP based on structural degradation. GWH-GLBP extract a new structural feature that calculate the gradient weighted histogram (LBP) of local binary mode on the gradient graph (GW-GLBP) to represent the image content. The complex degradation mode caused by multiple distortion is described effectively by the model; Wu et al. [26] believed that traditional structural descriptors only described the strength characteristics of structures, but could not effectively represent the spatial correlation of structures. Therefore, they introduced a model based on directional selectivity to represent the spatial correlation of structures. Then, a new structure descriptor is proposed according to the gradient size and the pattern based on direction selectivity. Finally, the new structure descriptor is used to extract the image structure, and the structure histogram based on direction selectivity is established to represent the image content; Li et al. [27] proposed an NR-IQA algorithm called “NRSL” based on structure and luminance information. The model utilized two statistical distributions on normalized luminance maps to characterize visual sensitive features of human eyes. First, the local contrast is normalized, and then the structure histogram and brightness histogram are extracted to represent image quality; Fang et al. [28] proposed a NR-IQA method called “NRLT” based on perception characteristics which applied in the field of SCI (screen content images). First, the histogram of the luminance graph is used to represent the statistical luminance feature in the global range. Then, four filters with different directions are used to calculate the gradient image of the luminance image, and the LBP histogram features are extracted as the statistical texture features of SCIs in the global scope. Finally, SVR is used to train the quality prediction model, and the quality perception features are mapped to the visual quality of the image.

Some of the models described above rely on human subjective experiments and require a database of human subjective scores (MOS). In order to overcome this difficulty, there are some IQA model, which are not rely on human subjective fractional. Mittal et al. [29] proposed a “completely blind” NR-IQA model called “NIQE,” in which the features are constructed based on the “quality perception” features of the successful NSS spatial domain derived from the simple but highly regular NSS model. First, a multivariate Gaussian (MVG) model is used to fit these features. Then, the NSS feature of the test image and the NSS feature of the reference image are extracted, respectively, and two MVG models are obtained by fitting and summing, respectively. Finally, the model calculates the distance between two multivariate Gaussian models to represent the image quality; Zhang et al. [30] proposed a method called “IL-NIQE” on the basis of “NIQE.” In addition to the two features used in NIQE, this method also introduced three additional quality perception features. Further, instead of using the global MVG model, the test image is divided into blocks, and the feature vectors of each block are fitted into an MVG model, and then a local quality score is calculated. Finally, the method gathers local quality score to obtain the final image quality score.

Recently, some NR-IQA models based on deep learning have been proposed. Ma et al. [31] proposed a multitask end-to-end optimized deep neural network (MEON) for NR-IQA, which consists of a distortion recognition network and a quality prediction network. The model training process is divided into two steps: first, train a distortion-type recognition subnetwork. Then, from the output of the pretrained early layer and the first subnetwork, an improved stochastic gradient descent algorithm is used to train the quality prediction subnetwork. Finally, the quality prediction subnetwork is used to predict the image quality. This model uses the group maximum differentiation competition method, which proves the strong competitiveness of MEON in NR-IQA model; Zhang et al. [18] argued that manually designed features could not accurately quantify the distortion of SR images, and the complex mapping between features and image quality scores could not be well approximated by a simple regression model. Therefore, they propose an NR-IQA model based on deep learning and superposition regression. First, the model uses pretrained VGGNet to extract depth features from SR images. Then, the model builds a superposition regression framework to learn the depth features of the image and finally predict the image quality.

The above NR-IQA model based on artificially extracts the features of different fields, but it is not applicable to SR images and cannot comprehensively represent the content of SR images. In other words, not all features are suitable for the quality assessment task of SR images, and there may be irrelevant or redundant features. This problem usually results in a decrease in the performance and efficiency of the NR-SRIQA model, and the predicted scores of the model may show a low correlation with MOS. The research purpose of this paper is to reduce the length of image feature vectors by feature optimization for the features used by some of the NR-IQA models mentioned above, removing the irrelevant and redundant features of SR images, and finally improving the performance and efficiency of the NR-SRIQA model. Therefore, with the feature optimization is vital to SR-IQA, which not only improve the predictive ability of NR-SRIQA model but also show a higher correlation between the model prediction score and human subjective scores, and it is important to apply this method to the field of SR-IQA and to establish an SR-IQA model based on deep learning laid a solid foundation.

## 3. Methods

As mentioned above, the general NR-IQA model does not consider the particularity of SR images. To solve this problem, the features that were related to the SR images closely are collected and aggregated first, which is described in detail in section A. In addition, considering that not all features collected are related to SR images, a feature optimization framework based on feature selection is proposed to optimize the collected feature set, see sections B and C for specific implementation. The proposed framework of this paper is shown in Figure 1.

### 3.1. Feature Extraction

It is considered that the local contrast features of SR images convey structural information that is closely related to image perception, the combined statistics of gradient magnitude (GM) and Laplacian of Gaussian (LOG) [32] are first used to represent the structural information of SR images, and b and c in Figure 2 show the GM map and LOG map of SR image a. Since image gradient amplitude is an effective method to encode image local contrast information and human vision system is highly sensitive to it, this paper uses the method in [25] which called GW-GLBP to extract features about SR image gradient amplitude. Furthermore, the SR image's brightness feature, chroma feature, LMS color feature, and hue saturation feature should also be considered. Therefore, this paper uses the Luma, Chroma.

LMS and HS mentioned in [16] to represent them, respectively. Brightness features mentioned in [15] are also considered in this paper. Figures 3(b)–3(d) and 3(e) represent the MSCN map, LAB map, LMS color map, and hue saturation map, respectively. The luminance feature, chroma feature, color feature, and hue saturation feature used in this paper can be extracted from b, c, d, and e, respectively.

In [17], the image SR is to restore the high-frequency components of LR images, which means the SR image can be transformed into the DCT domain and the generalized Gaussian model can be applied to fit the DCT coefficients to quantify the SR image artifacts. Additionally, the spatial discontinuity of pixel intensity is closely relevant to the perception score of SR image, hence this paper applies principal component analysis (PCA) [17] to image blocks and uses corresponding singular values to describe the spatial discontinuity. In order to enrich the initial feature set, this paper also extracted the directional Log-Derivative based on MSCN coefficient used in [33]. In general, this paper extracted 10 categories of image features from different fields, including 470 features, as shown in Table 1.

### 3.2. Feature Ranking

To rank the 470 features, five feature ranking algorithms are adopted in this paper: 1: Lasso [34]. 2: Maximal information coefficient (MIC). 3: Random Forest (RF). 4. Ridge regression. 5: Recursive feature elimination (RFE). To address the randomness of the feature ranking, each feature ranking algorithm is applied 100 times. Taking feature ranking on CVIU-17 [17] database as an example, a feature importance matrix **R***i* with a dimension of 100*∗*470 was first obtained, as shown below

(5) $$\begin{array}{c} Ri=\left(\begin{array}{ccccc} 41 & 45 & \ldots & 245 & 265\\ 41 & 40 & \ldots & 234 & 384\\ \ldots & \ldots & \ldots & \ldots & \ldots \\ 40 & 299 & \ldots & 233 & 28\\ 45 & 41 & \ldots & 59 & 265 \end{array}\right). \end{array}$$

In the matrix **R***i*, there is a feature importance ranking for each row that ranked from large to small, and the number in **R***i* represents the feature index. For conveniently measure, with the total importance of each feature, the weight of the feature with the highest importance in a single order was set as 470; then, the weight decreased by 1, and the weight of the feature with the lowest importance in a single order was set as 1. Calculate the *i*th feature importance by the following formula:

(6) $$\begin{array}{c} I_{i}=\sum_{i=1}^{n}X_{i}Y_{i}, \end{array}$$

where *n* is the number of columns and *X*_*i*_ are the setting weight of feature importance, *Y*_*i*_ represents the number of times the feature index appears in column *i*, *I*_*i*_ represents the importance degree of the feature, and then the features are sorted according to the size of *I_i_*. The feature matrix **M***(i)* (0 < *i* < 6) is obtained by the above calculation.

### 3.3. Train Model

As mentioned in [33], one problem of feature selection is how to determine the number of features in the model. In this section, we will investigate the linear correlation between the number of features and PLCC to determine the optimal number of features for the model.

After the feature matrix **M ***(i)* is obtained, the feature columns in each feature matrix are successively added to the feature set **S ***(i)* according to the importance of features, and one feature is added each time. Considering the efficiency of the model, the number of features studied in this paper is less than 100. After each operation of adding feature columns, support vector machine (SVM) [23] was used to learn the feature and training a model to predict the SR images quality. During the training process, grid search was used to select the optimal parameters Gamma and C. This step was cycled for 50 times, and the PLCC median of 50 cycle iterations was taken as the evaluation standard.

### 3.4. The Best Model

From the previous section, we obtained the correlation between the number of features and PLCC.  Figure 4 shows that Lasso use 15 features to achieve the PLCC value of 0.970, and 62 features to achieve 0.974; Mic reached the PLCC value of 0.954 with only 17 features, and 0.966 with 95 features; RF reached the PLCC value of 0.975 with only 53 features and 0.977 with 97 features; the PLCC value of RFE method reached 0.97 with only 55 features and 0.973 with 100 features; and the Ridge method achieves the PLCC value of 0.973 with only 44 features and 0.975 with 100 features. So, the model_o_ with the best performance is the eigenmatrix training model obtained by RF.

## 4. Results

In this paper, the performance of the proposed model is compared with other NR-IQA models on CVIU-17 and on QADS [4], and the proposed feature optimization framework is also applied to QADS. The experimental implement remained consistent when comparing model performance: first, the SR image features are extracted and divided into 80% training set and 20% testing set.

Then, an SVR regression model, in which the testing set is used for parameter tuning, is used to obtain the optimal parameters C and Gamma by grid search. Finally, the predicted score and human subjective score were used to calculate the PLCC value on the testing set. This step is iterated for 50 times, and the PLCC median of 50 iterations is taken as the evaluation standard.

### 4.1. The Best Model on QADS and CVIU-17 via Optimization

In this paper, the features described in II-A are first extracted from CVIU-17 and QADS databases, respectively, and then these features are optimized by using the proposed framework. We ended up using 97 of RF ranked features on CVIU-17 and 83 of ridge ranked features on QADS.  Figure 5 shows the work done on the QADS.

This paper also visualizes the linear correlation between the image score predicted by the model on the test set and human subjective score, as shown in Figures 6 and 7 The results show that the proposed model has good generalization performance and can accurately predict the quality of SR images.

### 4.2. Performance Comparison

In this paper, the proposed model is compared with a model using all 470 features and with some traditional manual feature-based methods, of which Beron20 is the most recent feature selection-based method. The results are shown in Tables 2 and 3.

The models with the best performance are indicated in red in Tables 2 and 3. The results show that the proposed models are optimal, and the efficiency and performance of the model can be further improved by using the feature optimization framework. For example, in this paper, 97 features used in CVIU-17 and 83 features used in QADS surpass the model with 470 features in performance. This also indicates that most of the features used by the existing models contain many redundant features, which not only makes the model inefficient but also has a certain impact on the performance of the model. These problems can be solved effectively by using the proposed feature optimization framework. In addition, there are practical requirements that can be met by using the proposed framework, such as sacrificing a small amount of performance in pursuit of time efficiency.

### 4.3. Discussion

After the SR-IQA model is obtained, the correlation between each feature and SR image will be discussed in this section, to explore which features of the SR-IQA model are most important. The ablation experiment is conducted to determine which feature class is the most important in the optimal model and relevant to SR image most. Figures 8 and 9 show the precision loss of the model after deleting a feature class, respectively. By observing Figures 8 and 9, it is found that the model established based on QADS has the largest loss of model accuracy when Luma and PCA are removed, while the model established based on CVIU-17 has the largest loss of model accuracy when GW-GLBP and Chroma are removed. Luma features include those most relevant to SR images, and there is considerable evidence that several types of retinal neurons undergo an excitatory inhibitory process around the local center, thereby providing a band-pass response to the brightness of visual signals. These features can be regarded as basic NSS features related to the classical retinal processing model, so the Luma features can well capture the distortion information of SR images. Some studies have pointed out that since the spatial discontinuity of pixel intensity is closely related to the perception score of SR image in subject research, PCA can be used to represent this feature. In addition, SR images contain rich texture details, which can be perfectly captured by GW-GLBP and DCT. Therefore, these features are highly correlated with SR images. In addition, considering that SR images are basically color images, Chroma can capture the chromaticity features of the images, as shown in Figures 8 and 9.

The results show that Luma, Chroma, PCA, and GW-GLBP all provide necessary information for predicting SR image quality. In building the optimal model, only some common existing features are used in this paper, and some features may not be suitable for the SR IQA task. How to discover or propose some features related to SR in order to obtain higher model prediction performance is the focus of the future work.

## 5. Conclusion

In this paper, an SR image quality assessment model based on feature aggregation is proposed, and a feature optimization framework is proposed to optimize the aggregated features. First, the advanced NR-IQA model is screened out, and relevant features are extracted to establish the initial feature set, and then Model_a_ is established. In order to further improve the efficiency and performance of the model, three feature selection algorithms were used to rank the importance of features in the feature matrix, and the linear relationship between the number of features and PLCC was studied. Finally, the optimal feature algorithm and the optimal number of features were determined to build the best model. It is also found in this paper that the performance and efficiency of our model based on feature aggregation can be improved by feature optimization. Experimental results show the effectiveness of the proposed framework.

This research has some limitations, naturally. Perhaps the most noteworthy concern is how to determine the candidate features. If the candidate features are not correlated with SR images, the performance of final constructed model would be poor. Investigating this will be an interesting extension to the present research. Future studies could consider building an end-to-end deep SR-IQA model to solve this problem. [20].

## Figures and Tables

**Figure 1:** The framework of the proposed method.

**Figure 2:** (a) Original image, (b) GM map of the original image, and (c) LOG map of the original image.

**Figure 3:** (a) Original picture, (b) MSCN map of the original picture, (c) LAB map of the original picture, (d) LMS map of the original picture, and (e) HS map of the original picture.

**Figure 4:** The correlation of PLCC and feature number on CVIU-17.

**Figure 5:** The correlation of PLCC and feature number on QADS.

**Figure 6:** The predicted scores and subjective MOS on QADS.

**Figure 7:** The predicted scores and subjective MOS on CVIU-17.

**Figure 8:** Performance loss after delete one feature class on QADS.

**Figure 9:** Performance loss after delete one feature class on CVIU-17.

**Table 1:** All features.

Features	Features index
Luma	f1–f74
Chroma	f75–f154
LMS	f155–f228
HS	f229–f232
BRISQUE	f233–f236
GMLOG	f237–f276
GW-GLBP	f277–f326
DCT	f327–f353
PCA	f354–f428
PLD	f429–f470

**Table 2:** Performance compare on CVIU-17.

Models	Criteria			
	SROCC	KROCC	PLCC	RMSE
Model_o_	**0.974**	0.863	**0.977**	5.281
Model_a_	0.973	**0.865**	0.976	**5.170**
BLINDS-II	0.921	0.763	0.932	8.739
DIVINE	0.925	0.773	0.941	8.265
BRISQUE	0.918	0.758	0.933	8.724
GW-GLBP	0.961	0.834	0.965	6.414
Beron20	0.969	0.852	0.973	5.533

**Table 3:** Performance compare on QADS.

Models	Criteria			
	SROCC	KROCC	PLCC	RMSE
Model_o_	**0.968**	**0.855**	**0.971**	**6.852**
Model_a_	**0.966**	**0.853**	**0.968**	**7.069**
BLINDS-II	0.862	0.683	0.872	14.117
DIVINE	0.933	0.781	0.934	10.128
BRISQUE	0.928	0.774	0.932	10.437
GW-GLBP	0.926	0.780	0.929	10.649
Beron20	0.965	0.847	**0.968**	7.099

## Data Availability

Data used in this paper can be accessed up on request from the corresponding author.
